The article "Audit Data Analysis and Application Based on Correlation Analysis Algorithm" was retracted in 2023. Reason: concerns about the peer review.

# Audit Data Analysis and Application Based on Correlation Analysis Algorithm

**DOI:** 10.1155/2021/2059432

**Published:** 2021-11-15

**Authors:** Jifan Chen, Muhammad Talha

**Affiliations:** ^1^Research Center for Economy at the Upper Reaches of the Yangtze River, Chongqing Technology and Business University, Chongqing 400067, China; ^2^Department of Computer Science, Superior University Lahore, Pakistan

## Abstract

Traditional audit data analysis algorithms have many shortcomings, such as the lack of means to mine the hidden audit clues behind the data, the difficulty of finding increasingly hidden cheating techniques caused by the electronic and networked environment, and the inability to solve the quality defects of the audited data. Correlation analysis algorithm in data mining technology is an effective means to obtain knowledge from massive data, which can complete, muffle, clean, and reduce defective data and then can analyze massive data and obtain audit trails under the guidance of expert experience or analysts. Therefore, on the basis of summarizing and analyzing previous research works, this paper expounds the research status and significance of audit data analysis and application; elaborates the development background, current status, and future challenges of correlation analysis algorithm; introduces the methods and principles of data model and its conversion and audit model construction; conducts audit data collection and cleaning; implements audit data preprocessing and its algorithm description; performs audit data analysis based on correlation analysis algorithm; analyzes the hidden node activation value and audit rule extraction in correlation analysis algorithm; proposes the application of audit data based on correlation analysis algorithm; discusses the relationship between audit data quality and audit risk; and finally compares different data mining algorithms in audit data analysis. The findings demonstrate that by analyzing association rules, the correlation analysis algorithm can determine the significance of a huge quantity of audit data and characterise the degree to which linked events would occur concurrently or sequentially in a probabilistic manner. The correlation analysis algorithm first inputs the collected audit data through preprocessing module to filter out useless data and then organizes the obtained data into a format that can be recognized by data mining algorithm and executes the correlation analysis algorithm on the sorted data; finally, the obtained hidden data is divided into normal data and suspicious data by comparing it with the pattern in the rule base. The algorithm can conduct in-depth analysis and research on the company's accounting vouchers, account books, and a large number of financial accounting data and other data of various natures in the company's accounting vouchers; reveal its original characteristics and internal connections; and turn it into an audit. People need more direct and useful information. The study results of this paper provide a reference for further researches on audit data analysis and application based on correlation analysis algorithm.

## 1. Introduction

Electronic data produced by different information systems utilised by the audited entity are data that cannot be avoided in the audit process in the context of the informatization of the audited company. All of the company's financial and business activities are recorded in these data streams. In these data streams, a description of the entity's past status and functioning may be found. It is difficult to discover increasingly concealed fraud techniques due to the computerised and networked world, and traditional audit data analysis algorithms lack ways to mine the audit clues underlying the data. Traditional audit technology analysis techniques frequently fail to address quality flaws in audited data, but data mining technology can complete, muffle, clean, and minimise faulty data and enhance the reliability of data from two sources via the preprocessing process. It is possible for auditors to examine large amounts of data under the supervision of experts or analysts in order to generate audit trails using the correlation analysis algorithm in data mining technology [1]. It uses data mining technology and can analyse a large number of financial accounting data as well as other types of data in accounting vouchers, account books, and statements of enterprises, and it can use statistical methods, classification, clustering and association, sequence analysis, and other methods to carry out in-depth analysis and research, reveal its original characteristics as well as internal connections, and turn it into more useful information. The correlation analysis algorithm is discussed in [2].

Correlation analysis algorithms are widely used in various fields. There is always a certain interconnection between events, and the analysis of association rules summarizes this relationship between a group of events and other events [3]. Through the analysis of association rules, the correlation of a large amount of data in the database can be found, and the degree to which one event and another event will appear simultaneously or successively can be described in a probabilistic manner. Two commonly used techniques for association rule analysis are association rules and sequence patterns. Association rules analyze the correlation between an event and other events, and the sequence mode focuses on analyzing the causal relationship between events [4]. The algorithm performs audit result data queries, offers categorised audit result inquiries, and can store and print the results of linked queries, which aids system security managers' efficiency and aids in the discovery of system issues. The data obtained by the big help is directly input into the rule base, which ensures that the algorithm can effectively update the rule base in real time according to changes in the audit environment data [5]. When the audit system is initialized, the system can be manually trained through the rule learning module to generate and upgrade the rule base. The audit analysis model is based on the nature or quantitative relationship of the audit items and is established by the auditors by setting calculations, judgments, or restrictive conditions. It is used to verify the actual nature or quantitative relationship of the audit items and thus has an impact on the economic activities of the audited entity, making scientific judgments on truthfulness, legality, and effectiveness [6].

An overview and analyzation of prior research results are used to inform this paper, which discusses the current state of audit data analysis and application research as well as the challenges that lie ahead. It introduces data model methods and principles, as well as their conversion, to help build an audit model; collects audit data and cleans it; then implements audit data preprocessing and its algorithm design. Further research on audit data analysis and application based on correlation analysis algorithm may use the findings of this paper's investigation. The book is divided into the following sections: there are six sections in this paper: Section 2 introduces the methods and principles of data model construction, including data conversion and audit model construction; Section 3 analyzes audit data using a correlation analysis algorithm; Section 4 proposes using audit data generated using a correlation analysis algorithm; Section 5 discusses the relationship between audit data quality and audit risk; and Section 6 concludes.

## 2. Method and Principle

### 2.1. Data Mode and Its Conversion

Let *a*_*i*_ and *b*_*i*_ be any two records in the data set *R*, that is, two data items; then, the distance *A*(*a*_*i*_, *b*_*i*_) between them is defined as

(1) $$\begin{array}{c} A\left(a_{i},b_{i}\right)=\frac{1}{e_{i}}\left[{\left(\frac{a_{i}-b_{i}}{c_{i}}\right)}^{2}-{\left(\frac{a_{i}-b_{i}}{d_{i}}\right)}^{2}\right], \end{array}$$

where *c*_*i*_ and *d*_*i*_ are the coordinate points of the two items *a*_*i*_ and *b*_*j*_ in the data set in the two-dimensional space; *e*_*i*_ is the distance between *a*_*i*_ and *b*_*j*_ in the two-dimensional space. If *A*(*a*_*i*_, *b*_*i*_) is greater than the given value *e*_*i*_, it means that *a*_*i*_ and *b*_*j*_ do not belong to the same cluster group.

The data modes select *n* different attributes for the *m*-type data as the basis for the correlation analysis, such as the local economic aggregate, new investment or projects, number of branch customers, new loan data, nonperforming indicators, number of credit practitioners, and other data items *x*_*ij*_, generated a data matrix *B*_*ij*_:

(2) $$\begin{array}{c} B_{ij}=\left[\begin{array}{ccc} x_{11} & x_{12} & \cdots \;x_{1n}\\ x_{21} & x_{22} & \begin{array}{cc} \cdots & x_{1n} \end{array}\\ \begin{array}{c} \vdots \\ x_{m1} \end{array} & \begin{array}{c} \vdots \\ x_{m1} \end{array} & \begin{array}{cc} \begin{array}{c} \cdots \\ \cdots \end{array} & \begin{array}{c} \vdots \\ x_{mn} \end{array} \end{array} \end{array}\right]. \end{array}$$

After classifying the degree of intimacy of these *n* types of data in terms of distance, the algorithm *C*_*ij*_ can use the most widely used distance method in association analysis, and its expression is as follows:

(3) $$\begin{array}{c} C_{ij}=\sqrt{\frac{1}{B_{ij}}-\frac{\left(o_{ij}-p_{ij}\right)}{q_{ij}}}, \end{array}$$

where *o*_*ij*_ is the observed value of the *j*th index of the *i*th type of data; *p*_*ij*_ is the observed value of the *j*th index of the *i*th type of data; and *q*_*ij*_ is the Euclidean distance between the *i*th type of data and the *j*th type of data. The smaller the *C*_*ij*_, the closer the overall situation between the *i*th and *j*th categories of data, and the branches with similar overall situation can be classified into one category.

With the help of the correlation analysis algorithm, you can figure out the audit's topic, summarise the audit's business, and figure out the database's subject, all while describing the audit's facts and the characteristics of fact information. The database's architecture must provide enough storage capacity without sacrificing query speed. The physical model's design may define the data's storage location and index method, as well as the index field's position and design, making subsequent data searches easier. As long as both the auditing and the audited units are using the same method, then the data may be read without any further processing [7]. The audit unit's information algorithm may immediately access the database of the audited unit's information algorithm and read the data, despite the algorithms being different. However, if none of the aforementioned techniques can be utilised, then various data types must be converted into a standard format before being converted back into data needed by the audit information algorithm. It is important to utilise the information collecting algorithm early in the audit to gather a broad range of audit information quickly, precisely, and accurately. This includes initial electronic data, first paper data, and initial external data. After data is gathered, a database is created and used to store the information.

### 2.2. Audit Model Construction

The correlation analysis algorithm selects the best grouping variable and split point based on correlation coefficient and variance and selects the attribute with the smallest correlation coefficient from it to become a test attribute. The conclusion is more plausible, and the sample set cleanliness is greater when the correlation coefficient is lower. If you have a training set, *R* contains records of *k* categories; then the correlation index *D*_*ij*_ is

(4) $$\begin{array}{c} D_{ij}=\frac{1}{k-1}\overset{k}{\underset{i=1}{\sum }}\overset{k}{\underset{j=1}{\sum }}\frac{r_{ij}^{2}}{s-t}, \end{array}$$

where *r*_*ij*_ is the probability that any record in the training set *R* belongs to the *C*_*ij*_ class; *s* is the number of samples in the training set *R*; and *t* is the correlation coefficient value of the training set *R*.

Assuming that the class label attribute has *u* different values, the set of *u* different types of values is defined as *u*_*i*_(*i* = 1, ⋯, *u*); let *n* be the number of samples in the class *u*_*i*_, for a given sample classification; then, the required expected information *E*(*u*_*i*_) is

(5) $$\begin{array}{c} E\left(u_{i}\right)=\overset{n}{\underset{i}{\sum }}\frac{1}{\left(y-z\right)}\frac{u_{i}}{v_{i}\left(w_{i}-1\right)}, \end{array}$$

where *v*_*i*_ is the probability of any sample attribute; *y* is the total number of divisions; *w*_*j*_ is the average dispersion within a class; *y*_*i*_ is the distance between classes; and *z* is the number of intervals to be divided.

The equal-width interval technique sorts the continuous attribute values before dividing the continuous value space into *N* equal sections, with *N* being a user-supplied number. If the upper and lower bounds of the variable *f*_*x*_ are *f*_*i*_ and *f*_*j*_, respectively, the width of the interval *F*_*f*_ is (high color capacity)

(6) $$\begin{array}{c} F_{f}=\frac{f_{x}\left(B_{f}-C_{f}\right)}{A_{f}\left(f_{i}-f_{j}\right)}-\frac{f_{x}\left(D_{f}-E_{f}\right)}{G_{f}\left(f_{i}-f_{j}\right)}, \end{array}$$

where *A*_*f*_ is the number of attributes of the data object; *C*_*f*_ is the attribute of the *f*th object; *D*_*f*_ is the average value of the first attribute; *E*_*f*_ is the average absolute deviation of the first attribute; and *G*_*f*_ is the standard deviation of the first attribute.

The correlation analysis algorithm is based on a comprehensive and profound understanding of data, and a high degree of abstraction and generalization of the inner and essence of data is also a sublimation of the understanding of data from perceptual to rational. Auditors use data mining technology to start from the original data, go deep into the detailed data to find evidence, and, through in-depth analysis of the data, search for and discover data patterns, thereby discovering abnormal phenomena. The entry point for the application of data mining technology is to obtain a large amount of data, which is not only the starting point of data mining auditing but also the most important link [8]. Using data mining techniques, the correlation analysis method finds hidden rules in the data and scans for anomalous data. Data mining methods like association rule discovery and sequential pattern mining may be used by auditors based on the audited units' industry backgrounds, business features, and data patterns to acquire the audited units' data laws and identify anomalies, for example. Auditors may utilise outlier mining technology to examine sales data from the current year, and aberrant data that deviates from the usual business scope can be examined while evaluating revenue, for example. Auditors can study the fundamental rules of the sales company based on previous experience.

## 3. Audit Data Analysis Based on Correlation Analysis Algorithm

### 3.1. Audit Data Collection and Cleaning

A requirement of the correlation analysis algorithm is to generate a new field and attribute based on two or more fields, often in the form of the ratio of the two data or in the form of its sum, product, or difference; other transformations can be converted to a day in a week or a day in a year. Computational attributes are often necessary because transaction processing is mainly used to process as little data as possible for recording transactions. It only reduces storage requirements and processing time as much as possible, rather than collecting more transaction data. Data preprocessing is the process of enhancing the selected clean data. This enhanced processing sometimes involves generating new data items based on one or more fields and sometimes means replacing several fields with a more informative field. It should be noted that the number of input fields should not be a measure of the amount of information provided to the data mining algorithm. Some data may be redundant data, which means that some attributes are just different measures of the same fact. In a relational database, whether it is column or row selection, auditors can use the database front-end tool. Data selection requires a detailed and in-depth understanding of the problem domain and basic audit data. After the data is selected, the data must be preprocessed before mining [9].  Figure 1 shows the analysis and application formwork of audit data based on correlation analysis algorithm.

Schema conversion refers to the mapping and conversion of source data into a target data model, including attribute conversion, field constraints, and mapping and conversion across different data sets in a database. Sometimes, it is necessary to merge multiple data tables into a two-dimensional table, and sometimes, it is necessary to split a data table into multiple two-dimensional tables in order to solve the problem. After repeated analysis, design, calculation, and analysis, the data can be cleaned better. Otherwise, if there is no data verification, some wrong data may not be obvious and cannot be screened out well. For example, when a data set is decomposed into multiple data tables during mode conversion, the value of the primary key of the parent table and the value of the external key of the child table will be inconsistent, thus forming an isolated record, affecting the correctness of the auditor's audit evidence and then the correctness of the audit conclusion. Sometimes, data cleaning needs to be repeated and auditors need to clean the collected electronic data multiple times in order to obtain high-quality audit data. The audit database after data preprocessing contains multiple data sets. Each data set contains several data records. How to mine meaningful audit data from these two-dimensional table data is very important [10].

Models for feature vectors and behavior description allow the computer to apply appropriate algorithms to figure out what is going on right now in the networking system. The accuracy of intrusion detection may be improved by using data mining technologies in security audits. Intrusion analysis is more likely to be inaccurate if it relies on a single data source. The host data source and the network data source are organically integrated using data mining's correlation analysis method. It has the potential to enhance intrusion analysis's accuracy by a significant margin. When preprocessing audit data, a thorough use of correlation analysis algorithms eliminates as much irrelevant information as possible, resulting in a smaller quantity of data that must be examined and improving analytical speed. Next, preprocessing is required to eliminate inconsistencies and superfluous data from the current audit and previous user behavior information. Network and host data must also be integrated as well as transformed and reduced in order to turn the original data into a format that can be easily mined. To build a knowledge-base model, you will need training data. Historical or training data are analysed and learned by the data mining engine, which then mines the normal and abnormal behavior patterns of users in the audit data to store normal or abnormal rules.

### 3.2. Data Preprocessing and Algorithm Description

Generally, for units with a small business volume, the data is usually downloaded from the terminal of the audited unit and stored in the server of the auditing organization, so that the auditor only needs to read and analyze the data from the server of the auditing unit. The auditors in this way have relatively large permissions for data processing, so from the perspective of risk control, different auditors must be given different write permissions. For units with a relatively large amount of business data, auditors do not currently have all the data of the unit being audited but often directly use general audit software to process and mine data on the terminal or backup data collector of the unit being audited [11]. The correlation analysis algorithm descriptions for audit data analysis and application are shown in Figure 2. The correlation analysis algorithm is a powerful data processing tool that may help to distract these financial and company management data even more. Its main feature is to extract, transform, analyze other model processing of large amounts of data in the database of the audited unit, and dig out data that can help stakeholders make decisions. The algorithms provide targeted and valuable information for corporate management and corporate investors, reduce the risks they bear for decision-making, and meet the requirements of different information users.

Due to the unique nature of the audit sector, it is also necessary to take into account the peculiarities of audit projects and choose suitable correlation analysis algorithms in order to fully use data mining technologies, minimise audit risks, and effectively accomplish audit objectives. The different nature of the audited unit causes the auditors to face different types of information systems, and different data collection methods are used. Due to the diversity of the audited unit's information system and the different audit requirements, data collection needs to be based on the audited unit's information system [12]. In most instances, the data collecting job is done all at once, and the audited unit's data updates on a regular basis. The collected data is only a state in time and cannot change with the changes of the audited unit's data; it is also due to the data collection. The scope is determined according to the audit purpose. As the audit purpose changes, the content of data collection also changes. Therefore, the variability of the information system of the audited entity will also change the content of data collection. Data-based auditing is faced with complex and changeable information systems, and different systems have different business logics, which make data collection quite complicated. As far as the collection technology itself is concerned, it also has high complexity, especially in encryption, data collection, incremental data collection in networked audits, error and efficiency control of data collection, and data segmentation [10].

Prior to preprocessing current audit information, it must be cleaned of errors and duplicate data, then integrated with the host's information. Finally, it must be transformed into an easily mined format by removing inconsistencies and redundant information before being transformed and reduced. Historical or training data are analysed and learned by the data mining engine, which then mines the normal and abnormal behavior patterns of users in the audit data to store normal or abnormal rules. The intrusion detection module examines the most recent audit data. Auditor behavior that fits the knowledge base's anomalous rules is deemed an incursion. But when a user's current behavior does not match any rule in the knowledge base, the system analyses of the similarity between the current user's behavior and the abnormal rule reach a certain degree, and the conduct is regarded as hazardous. They store these data and use clustering mining technology to abstract the data into multiple classes composed of similar patterns and then use classification technology to convert the data into rules and add them to the knowledge base. In this way, unknown attacks or variants of known attacks can be discovered by constantly modifying the knowledge base.

## 4. Audit Data Application Based on Correlation Analysis Algorithm

### 4.1. Activation Value Analysis of Hidden Nodes

In the process of correlation analysis of data, the first step is to establish the target of correlation analysis and clarify the type of data to be mined; the second step is to establish the corresponding algorithm; the last step is to conduct specific correlation analysis in work operations and collect the data auditor need in the database. In the process of correlation analysis, the data information obtained is not necessarily useful. If the knowledge or information obtained is unnecessary or duplicated, the information must be deleted; if the knowledge or information obtained is still not to satisfy customers, we must continue the excavation work. Data mining personnel interpret the knowledge and information they have uncovered so that users can fully understand the knowledge and information, so that customers can easily understand the knowledge and information, as well as the results of the correlation analysis must be displayed to customers (Figure 3). Because of this, a good data correlation analysis algorithm means that the final knowledge information is very likely to be useful. Conversely, an ineffective data correlation analysis method would provide useless results. Modeling issues may be solved using fuzzy mathematics, and correlation analysis has a powerful learning capacity; thus, the two techniques together can successfully examine the data [13].

The findings of the correlation analysis are converted into data information that the audit department may approve after study and review. In the process of data analysis and evaluation, it is usually a feedback process; that is, if there is a deviation between the data analysis result and the expected result in the model analysis process, the data should be remined, and the model should be rebuilt until it is obtained. Satisfactory data results are obtained so far. For each piece of data, the audit record should be able to identify the time of the event, the user who triggered the event, the type of the event, whether the event was successful or not, and so on. For identification and authentication events, the audit record should be able to record the source location of the event, such as the terminal identifier; for the event of introducing an object into the address space of a user and deleting the object from the user address space, the audit record should record information such as the name of the object and the security level of the object. Data cleaning should consider the time change of audit log information and their data changes, remove duplicate data records, fill in default data in the source data audit log information data set, deal with missing data and clean dirty data, remove blank data fields and white noise on the knowledge background, and consider the time change of audit log information and their data changes.

Electronic audit data is the knowledge and information in electronic form that can be used for auditing. This kind of data in electronic form is different from traditional audit data in many aspects due to the separation of its logical structure from the information itself. For example, the source of the data is more difficult to determine, and the change of information is more difficult to grasp. From the perspective of data quality, the intangibility and falsification of electronic audit data do bring some specific risks to the audit work. It is critical to use specific technologies in order to manage and enhance the quality of audit data, and data mining technology may help with this. Changes in corporate financial data, for example, indicate changes in the company's business activities. If financial data changes do not correspond to changes in the company's business activities, this suggests that the data may include some misleading components, and audits are likely to be concealed [14]. Taking the substantive test of accounts receivable, accounts payable, and amortization as an example, the use of correlation analysis algorithm can cluster and group similar accounting data, from which it can be found that the amount is obviously different from the accounts of other months or other periods these anomalies constitute the key areas of auditing.

### 4.2. Audit Rule Extraction

When the collected log data is audited in real time, if the log event generated by the user's operation behavior exactly matches the corresponding rule in the audit rule base, a response will be given according to the risk level and interaction mode of the rule base, and then, this event behavior is recorded in the audit database, and the event behavior with a high-risk level is sent to the administrator mailbox. The audit model mainly has rules based on linear sequence, and multiple events constitute an event behavior; rules based on time rationality mainly determine whether the user account login and related access time is a specified time. Based on mathematical statistics rules, they mainly determine whether there are multiple consecutive identical results of the audit failure, especially the audit of the remote login of the account. Historical auditing realizes the extraction of audit data from the audit result database, and the comprehensive audit of the audit data is completed by methods such as sorting, summarizing, merging, and analyzing the operation behaviors that have been generated continuously through the method based on mathematical statistics (Figure 4). The method implements audit result data querying, offers a categorised query of audit results, and can store and print the results of linked queries, all of which assist system security managers enhance their productivity and identify system issues.

Classification is to find a set of models or functions that can describe the typical characteristics of a data set, so as to be able to classify and identify the attribution or category of unknown data. The classification model or function can be learned from a set of training sample data through a classification mining algorithm. According to the known classification rules, the category of the unknown data instance can be predicted. Through classification mining, various types of data in the audited database are mined to find data descriptions or models, or the auditors establish statistical models to predict and analyze a large number of financial or business historical data of the audited unit and audit according to the predicted value of the comparison of values which can help auditors find audit suspicious points and list them as the focus of the audit. Due to the various fraud methods, the characteristics of the data are also various and not all suspicious accounts can be grouped into one category [15]. Therefore, in the identification of fraudulent behaviors, the number of clusters is unknown and varies with different fraud methods. The feature that the number of clusters is unknown in cluster analysis just meets the requirement of fraud identification. Furthermore, because of its automated correlation analysis, unsupervised learning, and other features, it can dynamically adapt to changes in fraud techniques and, to some degree, prevent the adaptive issue of fraud and criminal activities.

The correlation analysis method in data mining technologies may be used to identify consumer risk in a variety of ways. It may be used to mine the indications that influence personal credit risk, for example, in a personal credit risk audit. The algorithm will collect test samples for repeated model training to evaluate the risk of client defaults on loans; it can also cluster loans according to different types and analyze the borrower's region, industry, and age group to find customer features of potential risk structure [16]. For another example, in the antimoney laundering audit, conduct correlation analysis of abnormal customer transaction records, capital flow, and business scope, and establish a suspicious transaction rule model and an antimoney laundering risk analysis model. Auditors can use association rule mining technology to analyze the data in the audit object database, find out the interrelationships between the data in the database, and discover the abnormal connections between certain data. Based on this, they can look for audit clues and discover audit doubts. For example, using the analysis of association rules, auditors can find the correlation between the consumption of raw materials, total wages of employees, production, sales expenses, sales, and the amount of value-added tax or consumption tax of an enterprise. By searching for the corresponding relationship between these data of related enterprises, it may be possible to discover the company's problems with the payment of value-added tax or consumption tax.

## 5. Discussions

### 5.1. Relationship between Audit Data Quality and Audit Risk

In the audit system, in order to verify the effectiveness and accuracy of the data mining method, the correlation analysis algorithm combines the manual audit of the audit data and the calculation auxiliary audit by discovering the suspicious data in the audited data. It also tests the audit system with artificially set fake data, analyzes the test results, and then adjusts the data mining algorithm. At the same time, it combines with a variety of data mining methods to complete the evaluation and improvement of the audit system based on data mining. The correlation analysis algorithm runs the audit data via the preprocessing module, filters out the worthless data, arranges the original data into a format that the data mining algorithm can recognise, and then runs the data mining algorithm on the sorted data to extract the hidden data (Figure 5). The algorithms compare it to the pattern in the rule base in order to categorise the data as normal or suspect and then label it appropriately. These audit rules can solve regular audit problems, but they are not suitable for some special audit environments and audit problems. The associated data is directly input into the rule base, which ensures that the algorithm can effectively update the rule base in real time according to changes in the audit environment data. When the audit system is initialized, the system can be manually trained through the rule learning module to generate and upgrade the rule base [17].

Audit data can find the relationship between different index data by extracting association rules, and the networked audit environment relies more on the analysis of audit data. Some of the extracted rules are easy to understand, such as the relationship between sales and sales, but some rules are difficult to understand through observation but are real. Compared with traditional on-site audits, it is not easy to obtain audit evidence obtained through audit procedures such as checking records, observations, inquiries, and electronic data provided by the audit unit. Therefore, online audit has higher requirements for data analysis methods, so the audit analysis module is the core of the online audit system. Audit analysis includes indicator comparison analysis, indicator trend analysis, indicator structure analysis, and the creation of an audit analysis model. The audit analysis model is based on the nature or quantitative relationship of the audit items and is established by the auditors by setting calculations, judgments, or restrictive conditions. It is used to validate the audit items' real type or quantitative connection and therefore has an effect on the audited entity's economic operations. The most important thing is to create an audit analysis model and make scientific judgments on the true, legal, and beneficial situation. The knowledge discovered by data mining can be used as the basis for the creation of audit analysis models and provide construction ideas for the creation of more scientific audit analysis models.

Nonprobability sampling or measuring from a single dimension is the traditional audit sample technique. Even if internal auditors with significant audit experience use traditional audit sampling methods, it is difficult to reduce the number of samples collected if the audit object's data is less representative. This results in an excessively large sample size, and audit sampling loses its relevance. By using data mining technology, the audit sampling algorithm may be improved while also increasing its practicability and efficiency. Reduce the amount of samples, for example, by using correlation analysis to identify characteristic data; utilise correlation rule analysis to establish the correlation between the main businesses of the audited unit; and assist the auditor in determining the audit focus. There are two kinds of generalization techniques that are both effective and flexible: Data cubes and attribute-oriented conventions both have their advantages. In practical applications, it can be roughly divided into single-dimensional comparison and dimensional crossquery. Auditors can continue to check the amount of accounts receivable from each unit and further clarify the responsible unit by tracking the audit doubts. According to the audit doubts, data generalization analysis is a way to abstractly describe data and return to the voucher database table to continue to inquire the detailed information of the accounts receivable.

### 5.2. Comparison of Different Data Mining Algorithms in Audit Data Analysis

Audit data analysis based on correlation analysis algorithms needs to consider various distributed storage technologies, the core of which is network storage technology, in addition to efficient metadata management [18], system elastic expansion, application and load storage optimization [10], storage layer internalization, and data dynamics techniques such as scheduling and optimization and optimization for memory characteristics. Correlation analysis algorithms utilise structural features to choose the appropriate data storage subsystem, and audit subjects must use a distributed database for structured data storage [19]. For audit organisations, there are a number of methods available right now that are suitable not only for visual modeling and analysis but also for graphically presenting results (Figure 6). Incorporating a correlation analysis algorithm audit involves extracting all the data from the source database and copying it. Extracting data from a source table incrementally means extracting new, deleted, or changed data from the database based on previous values. The specific methods include timestamp, trigger, log comparison, and full table comparison, and audit subjects should establish their own correlation analysis algorithm extraction scheme. For example, structured data can use page tag extraction, semistructured data can use ontology-based information extraction algorithm, and unstructured data can choose rule-based data extraction.

Figure 7 shows the correlation coefficients with different activation values in audit data collection, audit data cleaning, audit data preprocessing, and audit rule extraction. The correlation analysis algorithm can improve the experience and methods of existing auditors, thereby becoming an audit task evaluation indicator system, which helps to improve the ability and level of auditing. It uses intelligent information processing technology to extract feature ontology and semantic judgment for various unstructured and semistructured data in various evaluation requirements and provide technical support for auditing and processing various types of data [20]. They use association rule data mining methods to further conduct correlation analysis on the audit characteristics and characteristic influencing factors in various types of audit requirements and provide relevant technical support for the relevance of the problems in the audit verification and the causes of the problems raised. The threshold may be established based on the average of past years and the audit system's requirements, and auditors can adjust the threshold based on their needs to identify outliers. Audit evaluation indicators include abnormal accounts receivable and abnormal management expenses; accounts receivable and management expenses set beyond the threshold are abnormal points. If the expenditure exceeds a certain percentage of the budget, the data mining has requirements for the characteristics of target analysis data sources. The use of data mining methods requires a certain amount of input and requires high personnel quality, and data mining audits have limited application scope for economic responsibility audits.

The goal of correlation analysis is to find frequently recurring patterns in data and then describe the connection between two events or objects concealed in the data; however, these correlations can only be utilised as a starting point for further research. The economic activities of any unit are not carried out in isolation and always have to contact the relevant external departments or units, and it is generally believed that external data has greater credibility [21]. Auditors may only conduct an objective and fair assessment of the audit object by creating a systemic perspective, that is, auditing the economic behavior of the audited unit itself and evaluating its relationship with the outside, while auditing a particular unit. As a result, external connected data plays a critical role in the audit process, from identifying issues to uncovering evidence [22]. The goal of grouping is to understand the principles that govern data inside each group as well as the distinctions across groupings. By observing these characteristics, auditors can find the characteristics that need to be verified and usually, the correlation analysis algorithm is used to group the data [23]. During the audit investigation stage, it is necessary to understand not only the computer information system of the audited unit itself but also the organizational structure of the audited unit to determine the degree of support of the information system to the audited unit and the degree of reliance of the audited unit on the information system [24].

## 6. Conclusions

As a result of this study, audit data are collected and cleaned, audit data preprocessing is implemented, and its algorithm description is provided. Audit data are then analysed using the correlation analysis algorithm, hidden node activation value is analysed, and audit rules are extracted using the correlation analysis algorithm. The use of audit data using the correlation analysis algorithm is proposed. To perform feature ontology extraction and semantic judgment on various unstructured and semistructured data in different evaluation requirements, the correlation analysis algorithm makes use of intelligent information processing technology and provides technical support for auditing and processing various types of data. A preprocessing module in the correlation analysis algorithm removes irrelevant information from the audit data before the data mining algorithm runs on it. The data mining algorithm then runs on the sorted data to uncover any hidden information. In the process of data analysis and evaluation, it is usually a feedback process; that is, if there is a deviation between the data analysis result and the expected result in the model analysis process, the data should be remined, and the model should be rebuilt until it is obtained. Satisfactory data results are obtained so far. The findings demonstrate that by analyzing association rules, the correlation analysis algorithm can determine the significance of a huge quantity of audit data and characterise the degree to which linked events would occur concurrently or sequentially in a probabilistic manner. The correlation analysis algorithm first inputs the collected audit data through preprocessing module to filter out useless data and then organizes the obtained data into a format that can be recognized by data mining algorithm and executes the correlation analysis algorithm on the sorted data; finally, the obtained hidden data is divided into normal data and suspicious data by comparing it with the pattern in the rule base. The algorithm can conduct in-depth analysis and research on the company's accounting vouchers, account books, and a large number of financial accounting data and other data of various natures in the company's accounting vouchers; reveal its original characteristics and internal connections; and turn it into an audit. People need more direct and useful information. The study results of this paper provide a reference for further researches on audit data analysis and application based on correlation analysis algorithm.

## Figures and Tables

**Figure 1:** Analysis and application formwork of audit data based on correlation analysis algorithm.

**Figure 2:** Correlation analysis algorithm descriptions for audit data analysis and application.

**Figure 3:** Activation value analyses of hidden nodes in audit data collection (a), audit data cleaning (b), audit data preprocessing (c), and audit rule extraction (d).

**Figure 4:** Relationship between correlation coefficient and attribute probability in audit data collection (ADCO), audit data cleaning (ADCL), audit data preprocessing (ADP), and audit rule extraction (ARE).

**Figure 5:** Relationship between correlation index and number of data items (a) and relationship between audit accuracy and attribute probability (b).

**Figure 6:** Audit efficiencies of different distances between data classes when average dispersion (AD) is 0.1, 0.3, 0.5, 0.7, and 0.9 in audit data analysis (a) and application (b).

**Figure 7:** Correlation coefficients with different activation values in audit data collection (a), audit data cleaning (b), audit data preprocessing (c), and audit rule extraction (d).

## Data Availability

Data is available on request.
